The article "Hydroxysafflor Yellow A Promoted Bone Mineralization and Inhibited Bone Resorption Which Reversed Glucocorticoids-Induced Osteoporosis" was published in 2018. Journal: Biomed Res Int.

# Hydroxysafflor Yellow A Promoted Bone Mineralization and Inhibited Bone Resorption Which Reversed Glucocorticoids-Induced Osteoporosis

**DOI:** 10.1155/2018/6762146

**Published:** 2018-07-05

**Authors:** Li Liu, Weiwei Tao, Wenjia Pan, Li Li, Qiong Yu, Dawei Zhang, Jun Jiang

**Affiliations:** ^1^School of Pharmacy, Guangdong Medical University, Dongguan 523808, China; ^2^Center for Translational Systems Biology and Neuroscience, School of Basic Biomedical Science, Nanjing University of Chinese Medicine, Nanjing 210023, China; ^3^School of Pharmacy, Jiangsu University, Xuefu Road, Zhenjiang, Jiangsu 212013, China

## Abstract

Glucocorticoids intake is the most common cause of secondary osteoporosis. Clinical studies have shown that 50% patients develop glucocorticoids-induced osteoporosis (GCIOP) after taking glucocorticoids for more than 6 months. Hydroxysafflor yellow A (HYA) is one main active ingredient in* Carthamus tinctorius *L. Previous studies have shown that HYA promoted bone marrow mesenchymal stem cells to differentiate into osteoblasts which promoted bone formation. Therefore, we speculated that HYA has a therapeutic effect on GCIOP. However, there is no in vivo evidence about the anti-GCIOP effect of HYA. In this paper, the effect of HYA (0.1, 1.0, and 10.0 *μ*M) on bone formation in normal zebrafish was investigated firstly. Secondly, the reversal effect of HYA on GCIOP was also evaluated by zebrafish model. It is demonstrated that HYA not only promoted bone formation in normal zebrafish (compared to* Control* group), but also reversed glucocorticoid induced bone loss (compared to* Prednisolone* group) according to the intervention of HYA in upregulating the area of mineralized bones (*p* < 0.01), increasing cumulative optical density (*p* < 0.01), promoting bone formation related gene expression (AKP, Type I, Runx2, OPG, and OCN,* p* < 0.01), inhibiting bone resorption related gene expression (TRACP,* p* < 0.01), and elevating whole-body trace mineral elements (Ca, P, K, Mg, Zn, and Fe) levels (*p* < 0.01). In conclusion, HYA had the potential to prevent and heal GCIOP by promoting bone mineralization, osteoblasts viability, and bone collagen expression and inhibiting bone resorption.

## 1. Introduction

Osteoporosis is a disease characterized by microarchitectural deterioration of bone tissue and decreased bone mass, leading to improved bone fragility and the increased risk of fracture [1]. The global population affected by osteoporosis is approximately 100 million, and it is about 69.4 million in China [2, 3]. Osteoporosis can be divided into primary and secondary type. Glucocorticoids intake is the most common cause of secondary osteoporosis [4, 5]. Glucocorticoids are very effective at treating human inflammatory and immunosuppressive effects. However, clinical studies have shown that, for patients taking glucocorticoids for more than 6 months, 50% develop osteoporosis [6, 7]. Furthermore, the incidence of fracture within such groups is approximately 30% after 5 years of treatment [8]. Thus, osteoporosis is a major limiting factor in the usage of glucocorticoids, even if patients are coprescribed bisphosphonates [9]. Related study has reported that glucocorticoids aggravated the aged osteoporotic status and impairment of skeletal metabolism [3] and thus increase the morbidity of osteoporosis and the risk of osteoporosis-related fractures. In vivo studies have shown that glucocorticoids treatment causes a decrease in bone formation through the suppression of osteoblasts in mice [10, 11]. Treatment with the glucocorticoids suppressed the number, activity, and differentiation of osteoblasts during ontogenetic growth, homeostasis, and regeneration of zebrafish bone [12].

The article "Hydroxysafflor Yellow A Promoted Bone Mineralization and Inhibited Bone Resorption Which Reversed Glucocorticoids-Induced Osteoporosis" was published in 2018. Journal: Biomed Res Int.

*Carthamus tinctorius *L. contains flavonoids, chalcones, alkaloids, and other chemical components and is a useful herb in painful osteoporosis [13]. Hydroxysafflor yellow A (HYA) is the main active ingredient of* Carthamus tinctorius *L. HYA prevented glucocorticoids-induced avascular necrosis of femoral head by inhibiting primary bone marrow mesenchymal stem cells (BMSCs) adipogenic differentiation [14]. In adults, BMSCs differentiate mainly into osteoblasts and adipocytes in the skeleton. Therefore, we firmly believe that HYA could be applied to cure osteoporosis, especially the glucocorticoids-induced osteoporosis (GCIOP).

Many animal models have been successfully used in GCIOP with different times of onset, including rat [15, 16], rabbit [17, 18], sheep [19], beagles [20], ewes [21], and pigs [22]. In the last decades, zebrafish has been affirmed as a powerful animal model [23, 24] to study bone development. Since the skeletal development of zebrafish has a high degree of similarity to human skeletal development, it is widely used. The zebrafish larvae treated with prednisolone as the model of GCIOP have shown a significant delay in early bone mineralization and regeneration [25].

In present work, we examined the effect of HYA on bone formation in normal zebrafish. And then, the zebrafish larvae were exposed in prednisolone (PNSL) to replicate the GCIOP model which was used to evaluate the therapeutic effects of HYA on GCIOP. Skeleton staining, bone formation/resorption related gene expression, and the bone mineral contents of zebrafish were carried out to assess the anti-GCIOP role of HYA in promoting bone formation and inhibiting bone resorption

The article "Hydroxysafflor Yellow A Promoted Bone Mineralization and Inhibited Bone Resorption Which Reversed Glucocorticoids-Induced Osteoporosis" was published in 2018. Journal: Biomed Res Int.

## 2. Materials and Methods

### 2.1. Ethics Statement

Animal experiments were carried out in accordance with the Guide lines for Animal Experimentation of Jiangsu University (Zhenjiang, China) and the protocol was approved by the Animal Ethics Committee of this institution.

### 2.2. Feeding Zebrafish

Zebrafish embryos were generated by natural mating and reared in 6 well plates containing blank E_3_ medium (5 mM NaCl, 0.17 mM KCl, 0.33 mM CaCl_2_, and 0.33 mM MgSO_4_). Embryos and larvae were maintained on a 14 h/10 h light/dark cycle and at a water temperature of 28.5°C [26].

### 2.3. Treatment Regime

At 2 days after fertilization (dpf), newly hatched zebrafish larvae were placed into 6 well plates (n = 15 larvae in each well) containing blank E_3_ medium 3 mL. Subsequently, the larvae were divided into different groups including Control (CON, blank E_3_ medium), prednisolone (PNSL, 25 *μ*M), disodium ethydronate (DE, 15 *μ*M DE and 25 *μ*M PNSL), and HYA (0.1, 1.0, or 10.0 *μ*M and 25 *μ*M PNSL) on 3 dpf. From 6 dpf to 10 dpf, larvae were fed with paramecia for 1 h every day. Following each feeding, the remaining paramecia were washed out and the medium was replaced with blank E_3_ medium containing drugs or not.

### 2.4. Skeletal and Matrix Staining

At the 10 dpf, all the zebrafish were killed by 3-aminobenzoic acid ethyl ester methanesulfonate (MS-222, 100 mg/L). After removal of MS-222 solution, zebrafish larvae were fixed in paraformaldehyde solution 4 % in PBS (pH 7.4) and stained with Alizarin Red S (ARS, 0.5 % KOH). 12 h later, adding fresh prepared bleach with 1.5 % H_2_O_2_ and 1 % KOH after the staining solution was removed and washed. 1 h later, all samples were decolored with glycerol and the stained zebrafish was placed under a microscope to observe their stained bones.

### 2.5. Bone Mineralization Analysis

Quantitative analysis of the area of mineralized bones (AMB) and cumulative optical density (COD) was performed as our previously described [27, 28]. Images of the ventral aspect of larvae skulls (ARS stained) were acquired using the Inverted fluorescence microscope (Olympus IX71/IX81, Olympus Corporation, Japan). Identical microscopic and camera settings were used for each treatment group. The AMB and COD were calculated using Image J software (National Institutes of Health, Bethesda, MD) for each treatment group (n=15).

### 2.6. RNA Isolation and Quantitative Real-Time PCR Analysis

Total RNA from larvae were isolated by Trizol (Ambion, Austin, TX), and cDNA was generated by reverse-transcription. Expression of AKP, type I collagen, Runx2, OPG, TRACP, and OCN were assessed by quantitative real-time PCR (Rt - PCR). Rt-PCR was performed on an ABI StepOnePlus TM real-time PCR system (one cycle of 95°C for 1 min and 40 cycles of 94°C for 10 s, 59°C for 30 s, followed by melt curve analysis). Relative expression was calculated using the formula 2^-ΔΔCT^. Primers used for PCR were listed in Table 1.

The article "Hydroxysafflor Yellow A Promoted Bone Mineralization and Inhibited Bone Resorption Which Reversed Glucocorticoids-Induced Osteoporosis" was published in 2018. Journal: Biomed Res Int.

### 2.7. Mineral Contents Detection

The mineral contents in zebrafish larvae were measured using inductively coupled plasma-mass spectrometry (ICP-MS) as our previous description [29]. The larvae were treated from 3 dpf to 10 dpf and collected at 10 dpf (n = 15 with three replications). The collected larvae were washed five times in double distilled water and then transferred to centrifuge tubes (10.0 mL). Immediately, samples were digested with 70 % HNO_3_ (Tama Chemicals, Kawasaki City, Japan) in a microwave oven for 4 h. Determination of Ca, P, K, Mg, Zn, and Fe was carried out by the 7500cx ICP/MS system (Agilent Technologies, Santa Clara, CA) equipped with a G3160B I-AS integrated autosampler.

### 2.8. Statistical Analysis

All data were presented as the mean ± SD. Differences were analyzed by one-way analysis of variance (Tukey/compare all pairs of columns). Statistical analysis was performed using GraphPad Prism 5 (GraphPad software, USA). Differences with* p* < 0.05 were considered significant.

## 3. Results

### 3.1. HYA Promoted Bone Mineralization in Normal Zebrafish

Bone mineralization is a stage of bone formation. Different concentrations of HYA (0.1, 1.0, and 10.0 *μ*M) were incubated with zebrafish in blank E_3_ medium (Figure 1(a)). Compared with the Control group, HYA significantly increased the area of mineralized bones (AMB,* p* < 0.01, Figure 2(a)) and cumulative optical density (COD,* p* < 0.01, Figure 2(b)). Bone formation related gene expression was examined in our research including AKP, type I collagen, Runx2, OPG, and OCN. HYA promoted the gene expression of AKP, Type I, OPG, and OCN (*p* < 0.01, Figure 3). Meanwhile, HYA inhibited the bone resorption related gene (TRACP) expression (*p* < 0.01). HYA had no significant effect on Runx2 expression. The whole-body Ca, P, K, Mg, Zn, and Fe levels were improved under the intervention of HYA (*p* < 0.01, Figure 4).

### 3.2. Glucocorticoids Decrease the AMB and COD in Zebrafish

AMB and COD are important indicators of bone mineralization. In our previous study, Alizarin Red staining was widely used to detect and quantify mineralized bones because it is capable of binding to calcium salts. We examined the optimal concentration of glucocorticoids (Prednisolone and Dexamethasone) in inhibiting bone formation (1.0, 2.5, 10.0, and 25 *μ*M). Treatment with Prednisolone at 25 *μ*M resulted in a significant decrease in AMB and COD compared to controls (Figure 1(b)).

The article "Hydroxysafflor Yellow A Promoted Bone Mineralization and Inhibited Bone Resorption Which Reversed Glucocorticoids-Induced Osteoporosis" was published in 2018. Journal: Biomed Res Int.

### 3.3. HYA Rescued the Inhibition of Bone Mineralization Caused by Glucocorticoids

HYA has good water solubility. In order to investigate whether HYA is able to attenuate the inhibition of bone mineralization induced by PNSL, three concentrations (0.1, 1.0, and 10.0 *μ*M) of HYA were applied from 3 to 10 dpf under 25 *μ*M PNSL treatment. Compared to the PNSL-treated group, AMB (Figure 2(a)) and COD (Figure 2(b)) values were significantly increased under the intervention of HYA (P < 0.01). This result indicated that HYA could rescue the inhibition of bone mineralization in zebrafish.

### 3.4. HYA Promoted Bone Formation Related Gene Expression and Inhibited Bone Resorption Related Gene Expression

Our results showed that 8 days (from 3 to 10 dpf) of PNSL treatment significantly reduced the expression of AKP, type I collagen, Runx2, OPG, and OCN (*p* < 0.01, Figure 3). After the treatment of HYA, the expression of these genes was significantly increased compared with the PNSL group (*p* < 0.01, Figure 3). On the contrary, HYA inhibited the expression of TRACP, a marker of bone resorption and reversed the elevation of TRACP induced by PNSL (*p* < 0.01, Figure 3).

### 3.5. HYA Promote the Enrichment of the Elements Required for Bone Mineralization

Bone was composed of 69-80 wt.% calcium phosphate and other components [30]. To confirm the therapeutic effect of HYA on osteogenesis, whole-body Ca, P, K, Mg, Zn, and Fe contents of larvae were measured by ICP-MS. Compared with the CON, the treatment of PNSL significantly decreased whole-body Ca, P, K, Mg, Zn, and Fe levels by 2.7-, 2.3-, 20.3-, 6.5-, 8.1-, and 8.8-fold, respectively (*p* < 0.01). After the treatment of HYA, whole-body Ca, P, K, Mg, Zn, and Fe levels were significantly higher than those in PNSL (*p* < 0.01, Figure 4). With the increase of HYA concentration from 0.1 to 10.0 *μ*M, the contents of these elements in zebrafish also showed an increasing trend and dose-dependence.

## 4. Discussion

In the theory of Chinese medicine,* Carthamus tinctorius* L. is considered to promote blood circulation and remove blood stasis, promote menstruation, and alleviate pain. Recent studies have found that* Carthamus tinctorius* L. is a useful plant in antiosteoporosis [31].* Carthamus tinctorius* L. contains different structural types of compounds including quinochalcones, flavonoids, alkaloids, polyacetylene, aromatic glucosides, and organic acids. Among them, HYA have been reported to be the major active compound with a content more than 13.24 g/kg [32]. In vitro studies have shown that HYA promoted the proliferation of human bone marrow-derived mesenchymal stem cells (BMSCs), induced BMSCs osteoblastic differentiation [33], and inhibited BMSCs adipogenic differentiation [14]. However, there is no in vivo study of HYA in antiosteoporosis. In this study, the antiosteoporosis effect of HYA in zebrafish model was first reported.

The article "Hydroxysafflor Yellow A Promoted Bone Mineralization and Inhibited Bone Resorption Which Reversed Glucocorticoids-Induced Osteoporosis" was published in 2018. Journal: Biomed Res Int.

The zebrafish model is a rapid, high content, in vivo model for glucocorticoids-induced osteoporosis studies. In this study, all of our experiments and data were finished and obtained within 15 days. The HYA used in this paper was isolated from* Carthamus tinctorius* L. extraction in our laboratory because it is difficult to obtain and high market price. Fortunately, this GCIOP model constructed from zebrafish does not need too much HYA. After calculation, the total amount of HYA used in this study was about 2 mg which is much lower than that of other in vivo organisms, especially rats.

This model is suitable for different kinds of natural compounds in the antiosteoporosis activity screening. Zebrafish absorbs drugs from the fish water either through the skin or gastrointestinal tract. If the compound is poorly water soluble, dimethyl sulfoxide (DMSO) may be chosen for solubilization. Zebrafish is DMSO tolerant, but the content of DMSO in the medium requires less than 0.5%. The water solubility of HYA is about 0.28 mg/mL at 25 °C [34]. But, prednisolone is a poorly water-soluble compound and DMSO is used for its solubilization. Therefore, in order to remove the interference caused by DMSO and make the administration of HYA more accurate, DMSO was also used in this study at the concentration 0.5%.

In the human body, bone is composed of calcium phosphate (69-80 wt. %, mainly hydroxyapatite), collagen (17-20 wt. %, mainly type I collagen), and other components (water, minerals, proteins, etc.). The collagen of bone was beneficial to the toughness (energy to fracture) of the bone, mitigating the brittleness of the mineral (Ca^2+^, Mg^2+^, K^+^, Zn^2+^, P, and others), and contributed to bone strength [13]. The mineral element concentration in zebrafish was in the order of Ca^2+^ > P > K^+^ > Mg^2+^ > Fe^3+^ > Zn^2+^. Treatment of HYA not only promoted the absorption of mineral elements, but also showed a double or triple (10.0 *μ*M) concentration of Ca and P higher than the DMSO group.

According to the literature, excessive Fe^3+^ exacerbates bone loss [35]. Our previous clinical study (117 postmenopausal women) also elaborated the serum ferritin (Fer) level which was significant negatively correlated with BMD (femoral neck and lumbar spine,* p* < 0.01). In addition, there was a significant positive correlation between serum Fer levels and serum PINP levels (*p* < 0.01). Serum Fer levels showed a significant positive correlation of serum *β*-CTX levels (*p* < 0.01). Therefore, postmenopausal Fe^3+^ overload exacerbated bone loss by promoting the degradation of type I collagen. However, all the zebrafish larvae used in this study were younger than 10 dpf which were in a stage where bone formation was greater than bone resorption [36]. Therefore, iron was an essential element involved in zebrafish larvae physiological functions. Glucocorticoids-induced iron concentration significantly decreases in zebrafish; HYA reversed the decrease in iron concentration (*p* < 0.01) and presented a dose-dependent manner from 0.1 to 10.0 *μ*M. This conclusion was consistent with the area of mineralized bones and cumulative optical density.

The article "Hydroxysafflor Yellow A Promoted Bone Mineralization and Inhibited Bone Resorption Which Reversed Glucocorticoids-Induced Osteoporosis" was published in 2018. Journal: Biomed Res Int.

AKP was secreted by osteoblasts and promoted bone mineralization. OCN is the dominant noncollagenous protein of the bone matrix. OPG is a decoy receptor that inhibits RANKL activation of osteoclasts, thereby decreasing bone resorption. Runx2 can directly stimulate the differentiation of bone marrow mesenchymal cells into osteoblasts. Moreover, AKP, OPG, and OCN were important indicators of osteoblasts activity. The expression of Runx2 reflects the ability of bone marrow mesenchymal stem cells to differentiate into osteoblasts. Tartrate resistant acid phosphatase, type 5b (TRACP), generally reflected the activity of the osteoclasts and the extent of bone resorption. Therefore, all the selected indicators AKP, OCN, OPG, RANK, Runx2, and TRACP are capable of responding to bone resorption and bone formation activity [37].

## Figures and Tables

**Figure 1:** Ventral view of Alizarin Red stained zebrafish skull at 10 dpf (×100). (a) Exposure to blank E3 medium and the effect of HYA on bone mineralization.** SAM**, the structure of zebrafish bones after staining;** CON**, blank E_3_ medium;** DE**, 15 *μ*M disodium ethydronate;** HYA 0.1**, 0.1 *μ*M HYA;** HYA 1.0**, 1.0 *μ*M HYA;** HYA 10.0**, 10.0 *μ*M HYA. (b) Exposure to prednisolone and the therapeutic effect of HYA on GCIOP.** CON**, blank E_3_ medium;** DMSO**, blank E_3_ medium + 0.5% DMSO;** PNSL**, blank E_3_ medium + 0.5% DMSO + 25 *μ*M prednisolone;** DE**, 15 *μ*M disodium ethydronate + PNSL;** HYA 0.1**, 0.1 *μ*M HYA + PNSL;** HYA 1.0**, 1.0 *μ*M HYA + PNSL;** HYA 10.0**, 10.0 *μ*M HYA + PNSL.** Note**: areas of calcified matrix in craniofacial skeleton are stained red.

**Figure 2:** The effect of HYA on mineralization in zebrafish larvae (n = 15). (a) Calculation of mineralized area. (b) Calculation of cumulative optical density.** Note**:** CON**, blank E_3_ medium;** DMSO**, blank E_3_ medium + 0.5% DMSO;** PNSL**, blank E_3_ medium + 0.5% DMSO + 25 *μ*M prednisolone;** DE**, 15 *μ*M disodium ethydronate;** DE+G**, 15 *μ*M disodium ethydronate + PNSL;** 0.1**, 0.1 *μ*M HYA;** 0.1 + G**, 0.1 *μ*M HYA + PNSL;** 1.0**, 1.0 *μ*M HYA;** 1.0 + G**, 1.0 *μ*M HYA + PNSL;** 10.0**, 10.0 *μ*M HYA;** 10.0 + G**, 10.0 *μ*M HYA + PNSL. ^#^Compared with CON,* p* < 0.01. ^ΔΔ^Compared with CON,* p* < 0.01. ^*∗*^Compared with PNSL,* p* < 0.05. ^*∗∗*^Compared with PNSL,* p* < 0.01.

The article "Hydroxysafflor Yellow A Promoted Bone Mineralization and Inhibited Bone Resorption Which Reversed Glucocorticoids-Induced Osteoporosis" was published in 2018. Journal: Biomed Res Int.

**Figure 3:** Effect of HYA on the expression of related genes in osteoporotic zebrafish larvae (n = 15). mRNA levels of the AKP, type I collagen, Runx2, OPG, TRACP, and OCN genes were determined by quantitative real-time PCR.** Note**:** CON**, blank E_3_ medium;** DMSO**, blank E_3_ medium + 0.5% DMSO;** PNSL**, blank E_3_ medium + 0.5% DMSO + 25 *μ*M prednisolone;** DE**, 15 *μ*M disodium ethydronate;** DE + G**, 15 *μ*M disodium ethydronate + PNSL;** 0.1**, 0.1 *μ*M HYA;** 0.1 + G**, 0.1 *μ*M HYA + PNSL;** 1.0**, 1.0 *μ*M HYA;** 1.0 + G**, 1.0 *μ*M HYA + PNSL;** 10.0**, 10.0 *μ*M HYA;** 10.0 + G**, 10.0 *μ*M HYA + PNSL. ^#^Compared with CON,* p* < 0.01. ^ΔΔ^Compared with CON,* p* < 0.01. ^*∗*^Compared with PNSL,* p* < 0.05. ^*∗∗*^Compared with PNSL,* p* < 0.01.

**Figure 4:** Effect of HYA on the mineral contents in osteoporotic zebrafish larvae (n = 15).** Note**:** CON**, blank E_3_ medium;** DMSO**, blank E_3_ medium + 0.5% DMSO;** PNSL**, blank E_3_ medium + 0.5% DMSO + 25 *μ*M prednisolone;** DE**, 15 *μ*M disodium ethydronate;** DE + G**, 15 *μ*M disodium ethydronate + PNSL;** 0.1**, 0.1 *μ*M HYA;** 0.1 + G**, 0.1 *μ*M HYA + PNSL;** 1.0**, 1.0 *μ*M HYA;** 1.0 + G**, 1.0 *μ*M HYA + PNSL;** 10.0**, 10.0 *μ*M HYA;** 10.0 + G**, 10.0 *μ*M HYA + PNSL. ^#^Compared with CON, P < 0.01. ^ΔΔ^Compared with CON, P < 0.01. ^*∗*^Compared with PNSL, P < 0.05. ^*∗∗*^Compared with PNSL, P < 0.01.

**Table 1:** Primer sequences for quantitative real-time PCR.

**mRNA**	**Forward sequence (5' - 3')**	**Reverse sequence (5' - 3')**
AKP	CAGGCAAATCAGTGGGAATC	TTGGGCATGTCTGCATCA
Type I	CAGGAGCCCAGTGTTGAG	AGCCACCAGACATCTGAGGA
Runx2	GACTCCGACCTCACGACAA	CGTCCCGTCAGGAACATC
OPG	CACTGCACAGTCAGGAGGAA	TGCTTTCGATGACGTCTCAC
OCN	GGCGCTACCTGGACCACTG	GCCGTAGAAGCGCCGATAG
TRACP	GCCTTCCTTCTTATCTCCT	CCCAATCCCTACAAACCT

## Data Availability

The data used to support the findings of this study are available from the corresponding author upon request.
